# Biofabrication of streptomycin-conjugated calcium phosphate nanoparticles using red ginseng extract and investigation of their antibacterial potential

**DOI:** 10.1371/journal.pone.0217318

**Published:** 2019-06-10

**Authors:** Gitishree Das, Kwang-Hyun Baek, Jayanta Kumar Patra

**Affiliations:** 1 Research Institute of Biotechnology & Medical Converged Science, Dongguk University-Seoul, Goyangsi, Republic of Korea; 2 Department of Biotechnology, Yeungnam University, Gyeongsan, Republic of Korea; North Eastern Regional Institute of Science and Technology, INDIA

## Abstract

Conjugation of nanoparticles (NPs) with antibiotics for treating multidrug resistant pathogens has been enormously studied now a days. In the current investigation, calcium phosphate (CaP) NPs were produced by co-precipitation using red ginseng extract as the reducing agent and were conjugated to the antibiotic streptomycin to form streptomycin-conjugated NPs (CPG-S NPs). The CPG-S NPs antibacterial activity was evaluated in this study against eight plant and five foodborne pathogenic bacteria. The synthesized CPG-S NPs were characterized by UV-VIS spectroscopy, scanning electron microscopy (SEM), energy-dispersive X-ray spectroscopy, Fourier-transform infrared spectroscopy, X-ray powder diffraction, and thermogravimetric and differential thermogravimetric analysis. CPG-S NPs exhibited promising antibacterial activity against all eight plant pathogenic bacteria and three of the five foodborne pathogenic bacteria tested; the diameter of inhibition zones ranged between 9.74–16.95 mm and 9.82–15.84 mm, respectively. CPG-S NPs displayed 50–100 μg/mL of minimum inhibitory concentration and 100 μg/mL of minimum bactericidal concentration against the plant and foodborne pathogenic bacterial strains, respectively. Furthermore, the SEM image of bacteria treated with CPG-S NPs displayed cells with a ruptured cell wall and fewer cells compared to the SEM image of untreated control bacteria displaying uniform and intact cells. SEM confirmed that CPG-S NPs degraded the bacterial cell wall and membrane resulting in lysed bacterial cells. In conclusion, the results suggest that CPG-S NPs could be effectively utilized in formulating drugs to treat bacterial plant or dental diseases and in manufacturing dental products such as toothpaste, mouthwashes, and artificial teeth.

## Introduction

Nanotechnology is considered a promising area of science for solving various problems in the field of health care and medicine. A number of nanoparticles (NPs) have been synthesized and studied for their potential applications in various fields, including the biomedical, pharmaceutical, and food sciences. Among these, the calcium phosphates (CaPs) have been extensively studied throughout the last few decades for their role in bone and teeth mineralization, as well as in pathological calcifications [1–5]. Recently, nano-structured CaPs have been used in numerous applications ranging from use as fluorescent labels and non-viral gene and drug delivery vectors to use in biomimetic dentin remineralization, in dental implant coating, and in customized 3D-printed structures of bone augmentation [1, 3, 4, 6–13]. Due to their osteoconductive properties and comparison to the inorganic constituent of natural bone, they have been further utilized to improve the biocompatibility of acrylic bone cements, bone fillers, and bone tissue engineering scaffolds [1, 3, 4, 6–13]. Besides, CaPs are widely used in the industrial and technological fields as catalysts and catalyst carriers for chemical responses in the field of environmental sciences, in materials for long-term ultraviolet protection, and as ion conductors and sensors [4, 14]. Finally, they are efficiently utilized in column chromatography for the rapid fractionation of biomolecules and also act as low-cost adsorbents for the removal of organic and heavy metal contaminants [4]. CAP-NPs were also demonstrated to be used in drug delivery system, in the encapsulation of microRNAs for the therapeutic treatment of cardiac cells [15]. In summary, CaPs are of interest for many biomedical applications due to their good biocompatibility and bioactivity [16]. Depending on their proposed use, the synthesis of CaPs may include the use of modifying agents to modify particle size and crystallinity, reduce agglomeration, and add specific functionalities [3, 11, 17]. A major issue in the synthesis of NPs is the choice of a proper procedure; the green synthesis process has been extensively accepted for its ecologically benevolent and non-toxic properties. This process can replace large scale synthesis of NPs and is suitable for the synthesis of nano-materials destined for biomedical applications.

*Panax ginseng* Meyer, most commonly known as the ginseng, is a perennial plant of the Araliaceae family [18, 19]. It is a traditional medicinal plant widely used in China, the Republic of Korea, Japan, and other Asian countries [20, 21]. The medicinal value of ginseng lies in its multiple pharmacological functions exerting anti-aging, anti-cancer, anti-stress, anti-diabetic, antioxidant, and anti-inflammatory effects [18, 20, 22]. Its major principal and bioactive components are the ginsenosides; more than 180 ginsenosides have been isolated and reported in various pharmacological and pharmaceutical studies [20, 23]. The most important part of the plant is the root, which is utilized in various ways such as raw in traditional foods. Alternatively, root extracts are used for the preparation of different tonics, health drinks, and health busting tablets [24]. Besides, a lot of ginseng products are available in market in the form of cosmetics and personal care products [24]. Considering the broad uses of the ginseng, CaPs were synthesized in this study using red ginseng root extract commercially available in the market and were conjugated with the antibiotic streptomycin. Furthermore, their antibacterial activity against both foodborne and plant pathogenic bacterial strains was evaluated.

## Materials and methods

### Biosynthesis of calcium phosphate nanoparticles using the red ginseng extract

CaP NPs were synthesized using a slightly modified method of the co-precipitation method by Banik et al. [25]; calcium nitrate and di-ammonium hydrogen phosphate were used as the reactants and red ginseng extract as the reducing and stabilizing agent. The obtained NPs were named CPG. The red ginseng extract (6-year old Ginseng- based Red Ginseng Extract Plus, Daedong Korea Ginseng Co., Chungnam, Republic of Korea) was purchased from a local shop in the Republic of Korea and was kept in the refrigerator until use. It was diluted 40 times, and before use, the extract and all reagents were sterilized separately. Twenty-five milliliters each of Ca(NO_3_)_2_. 4H_2_O (19.51 mM) and (NH_4_)_2_HPO_4_ (11.94 mM, pH 10) solutions, kept previously at 80°C for 30 min, were mixed in a beaker and stirred continuously using a magnetic stirrer at 80°C for 7 min. Following, 50 ml of red ginseng extract were added slowly over 10 min using a separating funnel. The final mixture was sonicated for 30 min for stabilization. The resulting CPG NPs were purified by centrifugation at 10,000 rpm for 30 min at 20°C and washed 2–3 times in sterile distilled water. The sample was dried at low temperature (50°C) in an oven and the powder was kept in a glass vial until further use.

### Preparation of streptomycin-conjugated CPG NPs

For the conjugation of streptomycin to CPG NPs, a slightly modified method of the standard procedure by Rastogi et al. [26] was used. A stock solution of 10 mg/ml streptomycin sulfate was prepared and stored in a deep freezer (-20°C) until use. One milliliter of the antibiotic stock solution was added dropwise to 5 ml of washed CPG NPs, and the solution was sonicated for 30 min followed by continuous stirring for 18 h. The obtained streptomycin-conjugated CPG (CPG-S) NPs were isolated by centrifugation, dried, and stored at 4°C until further use.

### Characterization of CPG-Streptomycin NPs

The newly synthesized CPG-S NPs were characterized by UV-VIS spectroscopy, scanning electron microscopy (SEM), energy-dispersive X-ray spectroscopy (EDS), Fourier-transform infrared spectroscopy (FT-IR), X-ray powder diffraction (XRD), and thermogravimetric and differential thermogravimetric analysis (TG/DTG) using standard analytical procedures [27–30].

The synthesized CPG NPs and CPG-S NPs were detected using a UV–visible microplate reader (Infinite 200 PRO NanoQuant, TECAN, Mannedorf, Switzerland) by scanning the absorbance spectra in the range of 230–730 nm at a resolution of 1 nm. The surface morphology of the synthesized CPG-S NPs powder was analyzed using FE-SEM (S-4200, Hitachi, Tokyo, Japan). The elemental composition was measured using an EDS detector (EDS, EDAX Inc., Mahwah, NJ, USA) attached to the FE-SEM machine. FT-IR analysis of the CPG-S NPs powder was carried out in the range of 400 to 4000 cm^−1^ wavelengths using a Jasco 5300 FT-IR spectrophotometer (Jasco, MD, USA). The structural features of the synthesized CPG-S NPs were analyzed using an XRD instrument (X’Pert MRD model, PANalytical, Almelo, The Netherlands) with Cu Kα radians at 30kV and 40 mA at an angle of 2θ. The thermal properties of CPG-S NPs were studied using an SDT Q600 TGA machine (TA Instruments, New Castle, DE, USA) from 20°C to 1400°C at a ramping time of 10°C/min under a N_2_ atmosphere inside the heating chamber of the machine.

### Antibacterial activity of CPG-S NPs against plant and foodborne pathogenic bacterial strains

The antibacterial effect of CPG-S NPs was evaluated against eight different plant pathogenic bacteria namely *Pseudomonas syringae* (*P*. *syringae*) pv. tobacci (Pstab), *P*. *syringae* pv. tobacci 11528 (Pstab11528), *P*. *syringae* pv. tomato T1 (PstT1), *P*. *syringae* pathovar tomato DC3000 (virulent), *P*. *syringae* pathovar tomato DC3000 (avirulent), *P*. *syringae* pv. actinidiae (Kyu-10), *P*. *syringae* pv. actinidiae (Kyu-16), and *Xanthomonas smithii* pv. citri (Yu-1). Antibacterial activity was also tested against five different foodborne pathogenic bacteria namely *Bacillus cereus* ATCC 13061, *Escherichia coli* ATCC 43890, *Listeria monocytogenes* ATCC 19115, *Staphylococcus aureus* ATCC 49444, and *Salmonella Typhimurium* ATCC 43174. The standard disc diffusion method was used to assess antibacterial activity [30]. The plant pathogenic bacterial strains were grown at 28°C in King’s B media (KB media, 20 g proteose peptone no. 3, 10 mL glycerol, 1.5 g K_2_HPO_4_, and 1.5 g MgSO_4_ per 1 L solution), and the foodborne pathogenic bacteria were grown in nutrient broth media (NB media containing 1 g D-glucose, 15 g peptone, 6 g sodium chloride, 3 g yeast extract per 1 L solution). For the antibacterial assay, cultures grown overnight were used. The sample solution was prepared by dissolving the CPG-S NPs in 5% dimethylsulfoxide (DMSO, 2000 μg/mL) and sonicating the samples at 30°C for 15 min. One hundred micrograms of CPG-S NPs/filter paper disc were prepared and used for the assay. Discs added the standard antibiotic streptomycin at 100 μg/disc were used as positive controls, while discs added 5% DMSO were used as negative controls. The antibacterial potential of the CPG-S NPs was determined by measuring the diameter of inhibition zones after 24 h of incubation at 37°C.

### Minimum inhibitory concentration (MIC) and minimum bactericidal concentration (MBC)

The MIC and MBC of the CPG-S NPs were determined by the two-fold serial dilution method [31]. First, 400 μg of the CPG-S NPs was added to the initial tube containing 2 mL of KB media for plant pathogens and NB media for foodborne pathogens, and mixed properly; from these tubes, 1 mL of each mixture was transferred to the next tube containing 1 mL of only KB/NB media, followed by proper mixing. Again, 1 mL of these mixtures was transferred to the next tube, and this procedure was repeated till the concentration of the CPG-S NPs in the last tube was 3.12 μg/mL. The positive control tube contains 1 mL of KB/NB media. Next, 10 μL of the tested pathogenic bacteria was added to each set of tubes excluding the negative control tube (only media). After this process was repeated for all the tested pathogenic bacteria, all the tubes were properly mixed and incubated at 37°C overnight in a shaker incubator. After the incubation period, the lowest concentration of the CPG-S NPs that showed no visible growth of the tested pathogen as compared to the positive and negative controls was determined as the MIC for that pathogenic bacterium. For the determination of the MBC, the tube that showed the MIC for the pathogenic bacteria and the tube with the next higher concentration were selected and spread separately onto the KB/NB agar plates, followed by incubation for 24 h at 37°C. The concentration of the extract for which no bacterial colonies were observed on the KB/NB agar plates was defined as the MBC value for that pathogenic bacteria. Both the MIC and MBC values were represented as μg/mL.

### Antibacterial mode of action of the CPG-S NPs on the pathogenic bacteria

The mode of action of the tested CPG-S NPs on the pathogenic bacteria was investigated by SEM using the standard procedure [32, 33]. Different pathogenic bacteria were treated with 5% DMSO (control) or the CPG-S NPs. Prior to the experiment, the pathogenic bacteria were grown overnight in their respective KB or NB media, and then, they were divided into two sections in fresh media (control without CPG-S NPs and samples treated with CPG-S NPs), and further grown overnight at 37°C. Then, these cultures were centrifuged at 1000 *g* for 10 min, after which the pellet was washed slowly with 50 mM phosphate buffer solution (pH 7.2) and then mounted over the glass slides and fixed with 100 mL glutaraldehyde (2.5%). The specimen was then dehydrated using different concentrations of ethanol (50%–100%) and finally, the ethanol was replaced by t-butanol, and the samples were incubated at room temperature for 2 h. After the incubation period, the specimens were sputter-coated with platinum in an ion coater for 120 s and observed under SEM (S-4100, Hitachi, Japan) for any changes in the morphology.

### Statistical analysis

All the experimental results are expressed as the mean ± standard deviation and the experiments are repeated three times. One-way analysis of variance (ANOVA) and Duncan’s test at P < 0.05 was also carried out using the Statistical Analysis Software (SAS) (Version: SAS 9.4, SAS Institute Inc., Cary, NC, USA).

## Results and discussion

### Synthesis and characterization of CPG-S NPs

In the current research, CaP-NPs were synthesized by using the commercially available red ginseng extracts using the co-precipitation process. The ginseng extracts are a rich source of natural bioactive compounds with multiple pharmacological potential [18, 20, 22]; thus, it is assumed that these bioactive compounds in the ginseng extracts might have played a major role in the synthesis process, particularly in capping and stabilization of the synthesized CPG NPs. After their synthesis, the CPG NPs were conjugated with the antibiotic streptomycin for the formation of CPG-S NPs and both the NPs were further characterized with regards to their morphological and chemical nature (Figs 1–5). The preliminary detection and nature of the synthesized CPG NPs and CPG-S NPs was determined by the UV-VIS spectral analysis (Fig 1). The synthesized CPG NPs and CPG-S NPs showed absorbance peak maxima at 276 nm and 280 nm, respectively. Similar results were obtained by previous researchers [27]. The slight deviation in the absorbance maxima of CPG-S NPs might be due to the red shift caused by the conjugation of streptomycin to the CPG NPs [27].

**Fig 1:** UV-VIS spectra of the synthesized CPG-S NPs. (Inset: Red ginseng extract used as reducing agent in the synthesis of NPs and the synthesized CPG-S NPs).

Further, the synthesized CPG-S NPs were subjected to FE-SEM-EDS analysis (Fig 2). The results of the SEM images showed a rod-shaped form with irregular borders. The images showed the nano size of individual particles with a highly rough surface (Fig 2A). Similar results were obtained by Martinez et al. [34]. The elemental composition of the CPG-S NPs was estimated by the EDS detector and the result is shown in Fig 2B. The CPG-S NPs contained 25.45 wt% of Ca, 11.66 wt% of P, 39.53 wt% of O, 22.95 wt% of C, and 0.41 wt% of Na. Viswanathan et al [28] has also studied the EDX spectra of CaP NPs that showed similar results with higher percentage of Ca and P. The FT-IR spectra of the synthesized CPG-S NPs showed the peak points at 3322.53, 1600.63, 1412.16, 1022.06, 595.00, and 557.96 cm^-1^ (Fig 3). The band at 3322.53 cm^-1^ corresponds to the N-H stretching of the primary and secondary amines. The band at 1600.63 cm^-1^ corresponds to the C-C stretching of the aromatic rings. The band at 1022 cm^-1^ corresponds to the C-N stretching of the aliphatic amines group, and the bands at 595 and 557 cm^-1^ correspond to the C-Br stretching of the alkyl halides. The study reveals the presence of both primary and secondary aromatic amines, which may be accountable for the synthesis and stabilization of the CPG-S NPs and could have acted as the reducing agent in the synthesis process [27]. The results of the FTIR observation revealed that the developed CPG-S NPs contained both inorganic and organic molecules. The FTIR spectra data of the CPG-S NPs corroborate well with the earlier reported spectra of CP NPs [16, 25, 27].

**Fig 2:** (A) SEM image of the synthesized CPG-S NPs; (B) EDS spectra of the synthesized CPG-S NPs (inset: percentage of different elements present in CPG-S NPs).

**Fig 3:** FT-IR spectra of the synthesized CPG-S NPs.

XRD data were obtained to evaluate the phase composition and the purity of the synthesized CPG-S NPs, and the results were compared with standard JCPDS 9–432 indexed patterns assigned to apatite (Fig 4, inset)[28, 35]. The CPG-S NPs revealed a 2θ degree corresponding to (002), (210), (211), (112), (202), (130), (222), (213), and (004) planes as shown in Fig 4. The results obtained are similar to those of Brundavanam et al. [35] and Arsad and Lee [36]. To determine density of the CPG-S NPs, TG/DTG analysis was performed, and the results are presented in Fig 5. A total of 51.09% weight loss was observed in three different phases when the temperature of the CPG-S NPs was gradually increased from 20°C to 1250°C in controlled N_2_ gas in the TGA machine chamber. The first phase of weight loss was observed between 12°C and 250°C, with a weight loss of 10.15%. The second weight loss was 22.05%, observed between 250°C and 600°C. The third weight loss was 18.89%, observed from 600°C to 1250°C (Fig 5). A relatively distinct weight loss of approximately 32.20% occurred between 20°C and 600°C. The weight loss occurring in three different phases was due to the degradation of water molecules during the first phase (within 250°C), loss of the organic materials from the red ginseng extract used during synthesis in the second phase along with water and CO_2_ loss (within 600°C) and the third phase weight loss (within 1250°C) may have resulted from degradation of the residual compounds, crystallization reaction, and phase changes [37], thereby confirming the involvement of the bioorganic compounds in the red ginseng extract in synthesis, capping, and stabilization of the CPG-S NPs, which are degraded with an increase in temperature [38]. The opposite nature of the peaks at approximately 200°C and 400°C of the DT curve implied endothermic and exothermic changes, respectively [25]. The peak at 400°C signified the initiation of CO_2_ loss [16, 25]. The decomposition temperature and the crystallization onset temperature in case of TG analysis generally differs with respect to the synthesis methods of calcium phosphates [39].

**Fig 4:** XRD spectra of the synthesized CPG-S NPs (inset: XRD spectra of the standard copper).

**Fig 5:** TG/DTG spectra of the synthesized CPG-S NPs.

### Evaluation of the antibacterial potential of CPG-S NPs against plant and foodborne pathogenic bacteria

The results of the analysis of the antibacterial activity of the CPG-S NPs and free streptomycin against different strains of plant pathogens (seven strains of *P*. *syringae* and one strain of *X*. *smithii*) are presented in Table 1 and Fig 6. Among all strains, the CPG-S NPs were highly effective against the *P*. *syringae* pv. actinidiae (Kyu-10) pathogen, showing a zone of inhibition of approximately 16.95 mm and was least effective against the *X*. *smithii* pv. citri (Yu-1), with a zone of inhibition of 9.74 mm. These results are comparable with those of the standard antibiotic, streptomycin (10.19 mm to 17.10 mm of inhibition zones), which was used as the positive control. Similarly, in case of the foodborne pathogenic bacteria, the CPG-S NPs were highly effective against *E*. *coli* ATCC 43890, yielding a zone of inhibition of 15.84 mm and least effective against *S*. *aureus* ATCC 49444, yielding a zone of inhibition of 9.82 mm. CPG-S NPs did not display positive activity against both *L*. *monocytogenes* ATCC 19115 and *S*. *Typhimurium* ATCC 43174. Moreover, CPG-S NPs yielded 50–100 μg/mL of MIC and 100 μg/mL of MBC against both plant- and foodborne pathogenic bacteria. Conjugation of CPG NPs with streptomycin yielded promising antibacterial effects (Tables 1 and 2 and Figs 6 and 7) when compared to treatment with only streptomycin. In such a case, the use of antibiotics and the associated issues can be reduced. Previous studies have reported that antibiotic-conjugated NPs exhibit promising antibacterial activity against numerous pathogenic microorganisms [40–42]. The antibacterial potential of the CPG-S NPs might also be due to the presence of various bioactive compounds in the red ginseng extracts, used during synthesis. Recently, the use of antibiotics has increased, resulting in the development of multiple resistant bacterial pathogens that can survive and multiply in the presence of an antibiotic and thus development of an antibiotic-conjugated NPs, which are effective against pathogens has also prompted a reduction in the use of generally acceptable antibiotics; CPG-S NPs can help resolve these issues. The CPG-S NPs with low MIC and MBC are probably applicable in, for instance, the formulation of antibacterial drugs to treat dental diseases, in manufacturing dental products including tooth paste, oral cleaning liquids, and other dental products. Moreover, it could also be utilized in manufacturing drugs and fertilizers for treating plants. There are reports on the antibacterial effect of CaP-NPs against a number of pathogenic bacteria in both intrinsically and synergistically with a number of antibiotics [43] and the current study strengthen their claim. Some reports also highlighted the combination of silver and CaP NPs and their effect against pathogenic bacteria such as *Escherichia col*i and *Staphylococcus aureus* [44]. Taken all together it can be said that CPG-S NPs could be highly effective as an antibacterial agent against a number of pathogenic microorganisms.

**Fig 6:** Antibacterial activity of CPG-S NPs against the eight different plant pathogenic bacteria.

**Fig 7:** Antibacterial activity of CPG-S NPs against the five different foodborne pathogenic bacteria.

**Table 1:** Antibacterial activity of calcium phosphate nanoparticles synthesized using ginseng extract and conjugated with streptomycin against plant pathogenic bacteria.

Plant pathogens	CPG-S^1^	Streptomycin^1, 2^	DMSO (5%)	MIC (μg/mL)	MBC (μg/mL)
*Pseudomonas syringae* pv. tobacci (Pstab)	10.32±0.30^f^	11.49±0.46^ef^	0	100	100
*Pseudomonas syringae* pv. tobacci 11528 (Pstab11528)	14.61±0.61^bcd^	15.46±0.19^abc^	0	50	100
*Pseudomonas syringae* pv. tomato *T1* (PstT1)	14.82±0.44^bcd^	10.19±0.17^f^	0	100	100
*Pseudomonas syringae* pathovar tomato DC3000 (virulent)	12.50±0.22^def^	17.10±0.28^ab^	0	100	100
*Pseudomonas syringae* pathovar tomato DC3000 (Avirulent)	15.92±0.41^abc^	16.13±0.22^cde^	0	50	100
*Pseudomonas syringae pv*. *actinidiae (Kyu-10)*	16.95±0.12^ab^	16.76±0.40^ab^	0	50	100
*Pseudomonas syringae pv*. *actinidiae (Kyu-16)*	15.76±0.33^abc^	18.03±0.57^a^	0	50	100
*Xanthomonas smithii pv*. *citri (Yu-1)*	9.74±0.53^f^	11.02±0.20^ef^	0	100	100

1) Data are expressed as the mean zone of inhibition in mm ± SD. Values with different superscript letters are significantly different at *P*< 0.05.

2) Streptomycin at 100 μg/disc

DMSO was taken as the negative control

**Table 2:** Antibacterial activity of calcium phosphate nanoparticles synthesized using ginseng extract and conjugated with streptomycin against foodborne pathogenic bacteria.

Foodborne pathogenic bacteria	CPG-S^1^	DMSO (5%)	MIC (μg/mL)	MBC (μg/mL)
***B*. *cereus* ATCC 13061**	11.24±0.38^b^	0	100	100
***E*. *coli* ATCC 43890**	15.84±0.21^a^	0	50	100
***L*. *monocytogenes* ATCC 19115**	0±0^d^	0	0	0
***S*. *aureus* ATCC 49444**	9.82±0.30^c^	0	100	100
***S*. *Typhimurium* ATCC 43174**	0±0^d^	0	0	0

1) Data are expressed as the mean zone of inhibition in mm ± SD. Values with different superscript letters are significantly different at *P*< 0.05. DMSO was taken as the negative control.

### Antibacterial mode of action of CPG-S NPs on pathogenic bacteria

To investigate the potential mechanism of action of the effect of CPG-S NPs against both the plant and foodborne pathogenic bacteria, SEM images of the treated bacteria were obtained and their surface morphology was compared to that of the untreated control bacteria. The SEM images of both the plant bacteria and foodborne bacteria treated with CPG-S NPs together with the untreated bacteria are presented in Figs 8 and 9. Compared to the untreated bacterial cells that showed, regular, uniform, and intact cells (Fig 8A–8G), pathogens treated with CPG-S NPs displayed fewer cells with a ruptured and disrupted cell wall (Fig 8I–8P). Compared to healthy, intact, and uniform untreated control bacterial cells (Fig 9A–9C), the pathogens treated with CPG-S NPs (Fig 9D–9F) displayed highly disrupted and ruptured bacterial cells with irregular morphology. The results confirmed that the CPG-S NPs had potent effects on both types of pathogenic bacteria, thereby killing them either through member disruption after penetration into the bacterial cells or by rupturing the inner membrane. Another study reported that silver NPs disrupt the stability of lipopolysaccharides present in the outer cell membrane of the bacterial cell, thus increasing the permeability of the outer membrane and the peptidoglycan layer of the cell wall, which might have been recognized and captured by the antibiotics, followed by the action of the NPs conjugated with antibiotics on the pathogen [45, 46]. Hence, we presume the same situation in the present case, wherein the CPG-S NPs could have affected the lipid layer of the outer cell wall, leading to degradation of the outer membrane, thereby causing destruction of the bacterial pathogen. According to another hypothesis, bioactive compounds of the red ginseng extracts [18, 22] serve as capping and stabilizing agents in the synthesis of the CPG-S NPs together with the antibiotics; this could have affected the cell wall surface, thereby rupturing the cell membrane and lysing the vital cell organelles, exposing them to the extracellular environment and ultimately leading to the death of the bacterial cells.

**Fig 8:** SEM image of the untreated control bacteria (A,B,C,D,E,F,G,H) and the CPG-S NPs treated plant pathogenic bacteria (I,J,K,L,M,N,O,P). *P*. *syringae* pv. tobacci (Pstab) [A,I]; *P*. *syringae* pv. tobacci 11528 (Pstab11528) [B, J]; *P*. *syringae* pv. tomato T1 (PstT1) [C,K]; *P*. *syringae* pathovar tomato DC3000 (virulent) [D,L]; *P*. *syringa*e pathovar tomato DC3000 (Avirulent) [E,M]; *P*. *syringae* pv. actinidiae (Kyu-10) [F,N]; *P*. *syringae* pv. actinidiae (Kyu-16) [G,O]; *X*. *smithii* pv. citri (Yu-1) [H,P].

**Fig 9:** SEM image of the untreated control bacteria (A,B,C) and the CPG-S NPs treated foodborne pathogenic bacteria (D,E,F). *B*. *cereus* ATCC 13061 (A,D); *E*. *coli* ATCC 43890 (B,E); *S*. *aureus* ATCC 49444 (C,F).

## Conclusions

This study shows that red ginseng extracts could serve as an excellent source of reducing agents for the synthesis of CPG NPs, which, on being conjugated with streptomycin, resulted in potential antibacterial effect against both plant and foodborne pathogenic bacteria. The biological synthesis of CPG-S NPs was easy, eco-friendly, and scalable. The conjugation of NPs with antibiotics could hence serve as a potential tool against multidrug-resistant pathogenic bacteria and could help minimize the use of antibiotics. The effective antibacterial potential of NPs conjugated with antibiotics render them better candidates for the formulation of nanomedicines to treat plant pathogens and as better candidates in the formulation of various dental products and drugs to treat bacterial dental diseases.
